The article "The effects of the COVID-19 pandemic period on stock market return and volatility. Evidence from the Pakistan Stock Exchange" was retracted in 2025. Reasons: unreliable results or conclusions; concerns about the peer review; concerns about the authorship.

# The effects of the COVID-19 pandemic period on stock market return and volatility. Evidence from the Pakistan Stock Exchange

**DOI:** 10.1371/journal.pone.0295853

**Published:** 2024-04-16

**Authors:** Baixiang Wang, Muhammad Waris, Katarzyna Adamiak, Mohammad Adnan, Hawkar Anwer Hamad, Saad Mahmood Bhatti

**Affiliations:** 1 School of Management, Chuzhou Vocational and Technical College, Chuzhou, China; 2 UE Business School, University of Education, Multan Campus, Pakistan; 3 Institute of Management and Quality Sciences, University of Justice, Warsaw, Poland; 4 Business and Management Department, SBS Swiss Business School, Geneva, Switzerland; 5 Department of Accounting and Finance, College of Administration and Economics, Lebanese French University, Erbil, Kurdistan Region, Iraq; 6 Institute of Business and Management (IB&M), University of Engineering and Technology (UET), Lahore, Pakistan; 7 Graduate School of Business (GSB), Universiti Kebangsaan Malaysia, Bangi, Selangor, Malaysia; Jiangsu University, CHINA

## Abstract

The COVID-19 pandemic has emerged as a significant event of the current century, introducing substantial transformations in economic and social activities worldwide. The primary objective of this study is to investigate the relationship between daily COVID-19 cases and Pakistan stock market (PSX) return volatility. To assess the relationship between daily COVID-19 cases and the PSX return volatility, we collected secondary data from the World Health Organization (WHO) and the PSX website, specifically focusing on the PSX 100 index, spanning from March 15, 2020, to March 31, 2021. We used the GARCH family models for measuring the volatility and the COVID-19 impact on the stock market performance. Our E-GARCH findings show that there is long-term persistence in the return volatility of the stock market of Pakistan in the period of the COVID-19 timeline because ARCH alpha (ω_1_) and GARCH beta (ω_2_) are significant. Moreover, is asymmetrical effect is found in the stock market of Pakistan during the COVID-19 period due to Gamma (ѱ) being significant for PSX. Our DCC-GARCH results show that the COVID-19 active cases have a long-term spillover impact on the Pakistan stock market. Therefore, the need of strong planning and alternative platform should be needed in the distress period to promote the stock market and investor should advised to make diversified international portfolio by investing in high and low volatility stock market to save their income. This study advocated the implications for investors to invest in low volatility stock especially during the period of pandemics to protect their return on investment. Moreover, policy makers and the regulators can make effective policies to maintain financial stability during pandemics that is very important for the country’s economic development.

## 1. Introduction

The decline in financial markets following the onset of the COVID-19 pandemic bears resemblance to the Global Financial Crisis of 2007–09 [1]. However, it is crucial to acknowledge that the underlying causes of the Global Financial Crisis and the current Covid-19 situation differ. The Global Financial Crisis stemmed from the actions of market participants, lenders, and speculators, constituting an internal shock. These behaviors resulted in substantial debt accumulation and risk-taking, ultimately leading to the formation of a credit bubble [2]. In contrast, the Covid-19 pandemic is an external phenomenon with direct economic consequences [3].

Various international organizations have revised their growth projections in response to the COVID-19 pandemic and the subsequent implementation of widespread lockdown measures. The International Monetary Fund has downgraded its global growth forecast for 2020 from 6.3% to -3%. Similarly, the Organization for Economic Cooperation and Development (OECD) anticipates a 1.5% decline in global economic growth by 2020 due to the extensive and ongoing spread of the coronavirus. Therefore, the outbreak of the deadly COVID-19 disease presents an opportunity to assess its impact on the stock markets of affected nations, particularly Pakistan.

The Covid-19 pandemic has had a significant influence on stock markets worldwide. According to [4] that the global health crisis caused by the virus has resulted in widespread economic disruptions and uncertainties, leading to volatility and market declines in the Indonesia. One of the primary reasons for the impact on stock markets is the disruption in global supply chains and business operations [5]. Measures such as lockdowns, social distancing guidelines, and travel restrictions implemented to contain the virus have temporarily halted or reduced the capacity of businesses across various sectors [6]. Therefore, these measures have led to decreased revenues, earnings, and profitability for many companies, prompting investors to reassess their portfolios and sell stocks. Additionally, investor sentiment and confidence have been severely shaken due to the uncertainty surrounding the duration and severity of the pandemic [7].

It is important to note that the impact of COVID-19 on stock markets has not been uniform across all sectors and countries. Certain industries, such as technology, e-commerce, and healthcare, have experienced growth and increased demand as a result of the pandemic [8]. Conversely, sectors heavily reliant on travel, hospitality, and physical retail have faced significant challenges [9]. Moreover, the COVID-19 pandemic has caused profound disruptions in global stock markets [10]. According to [11], economic repercussions, supply chain disruptions, and uncertainties surrounding the virus have contributed to market volatility and declines in the commodity market in Pakistan. However, the impact has varied across sectors and countries. Therefore, monitoring and analyzing the ongoing effects of the pandemic on financial markets remains crucial for investors, policymakers, and market participants to investigation in the emerging economy especially in Pakistan.

The stock market volatility gives significance to the change in the business operations environment [12] and hence it is an interesting problem for the investigations and provides a significant research gap for investigation in emerging economy such as Pakistan. Specifically, the first aims of this study are to investigate how the COVID-19 pandemic has affected stock market return volatility in Pakistan. Therefore, this study uses the historical stock market data to examine the patterns and changes in volatility during the COVID-19 period. This study also utilized various quantitative techniques and models to measure and assess stock market volatility, such as GARCH models or other volatility forecasting approaches, but previous study has the insufficient methodological approaches to estimate the volatility in spite of measuring the linear relationship between them. The second objective is to investigate the news impact of the COVID-19 that may fluctuate the stock market return of Pakistan and also investigating the symmetric and asymmetric news impact. Thirds aims is to investigate the spillover impact of the COVID-19 on the stock market return and volatility. Moreover, this study also provides the new insight about the volatility pattern in Pakistan with uniqueness or similarities of the pandemic’s impact on stock market volatility with respect to existing literature.

This study makes several contributions to the existing body of knowledge and theory, also proving the great implications for the investors, policy makers and the legislators. First, this study provides empirical evidence on the specific effects of the COVID-19 pandemic on stock market return volatility in the Pakistan Stock Exchange. By analyzing historical data and market performance during the pandemic period, this study quantified the magnitude of the impact, identified key drivers, and established the statistical relationships between pandemic-related factors and market dynamics. This empirical evidence enhanced understanding of the pandemic’s influence on the stock market in Pakistan. Second, by focusing on the Pakistan Stock Exchange, the study provided valuable insights into the unique characteristics and dynamics of the market. The study uncovered the pandemic impacted the Pakistani economy, investor behavior, and specific sectors, offering context-specific knowledge that informed the decision-making at the national level. In this way, this study findings are particularly adding novelty in the existing literature related to the pandemic of COVID-19 that has long term consequences on the stock market return that raise the risk especially in the debt burden economies such as Pakistan and create the critical thinking point for policymakers, market participants, and investors operating in the Pakistani market. Third, the long-term volatility existence in the Pakistani stock market generates the several problems for the economy to sustain in lowest growth ratio. Therefore, the findings of the study provided guidance for risk management and investment strategies during periods of crisis. By understanding the factors that drove market risk during the pandemic, investors and financial institutions make more informed decisions about portfolio diversification, asset allocation, and risk mitigation.

The implications of the study contributed to a deeper understanding of the consequences of the COVID-19 pandemic on the Pakistan Stock Exchange, enabling stakeholders to make informed decisions and implement measures to mitigate risks and promote market stability. Our findings are useful for the investors and the policy makers also, policy makers make the policy for meeting the uncertain events fluctuation and the investors can meet the potential return on their investment by evaluating the risk volatility during crisis and pandemics. The regulators also make rules in the period of pandemics and crisis to enhance their position by providing incentives to the financial sectors as well as other contributors of the stock markets. Moreover, the study has practical implications for market participants, including investors, financial advisors, and fund managers. By analyzing investor behavior, sentiment, and trading patterns during the pandemic, the research offers insights into how individuals and institutions responded to the crisis. This knowledge can inform the development of best practices, guidelines, and recommendations for investors to manage risk and make sound investment decisions in similar high-risk environments.

The remaining paper is organized as section 2 discusses the literature review including the theoretical as well as empirical literature. The methodology with the data description is included in section 3. The results and their discussion are illustrated in section 4 and the conclusion recommendations with policy implications and limitation are discussed in section 5. Moreover, the future research suggestions are also discussed in section 5.

## 2. Literature review

### 2.1 Theoretical background

There are several theories that support the study in the context of the middle income and emerging stock market. Efficient market hypothesis (EMH) suggests that financial markets, including stock markets, quickly and accurately incorporate all available information into stock prices [13]. The Efficient market hypothesis (EMH) also suggested that the news of the crisis or pandemic creates the volatility in the market that leads to utilization of the information the investors from the surroundings and the result in decline the prices level. This point of the news impact and the utilizations of the information motivate this study to extract the gape of the COVID-19 period to investigate the news impact in the period of the high risk and also the study examine whether the PSX adhered to the principles of the EMH during the pandemic or whether there were deviations from market efficiency. Behavioral finance theory explores how psychological and behavioral factors influence investor decision-making and market outcomes. The study analyzes how investor sentiment, risk aversion, and herding behavior during the pandemic impacted stock market risk. Contagion theory states that shocks or disturbances in one market can spread to other interconnected markets. On the ground of the theory concept, this study investigates whether the pandemic-induced shocks in global financial markets had a contagion effect on the Pakistan Stock Exchange, leading to increased risk. The Portfolio theory, particularly Modern Portfolio Theory, emphasizes the importance of diversification and risk management in constructing investment portfolios [14]. The study can explore how investors adjusted their portfolios and investment strategies during the pandemic to manage volatility, and the impact of these actions on the overall market dynamics. Moreover, by employing these theories and frameworks, the research can provide a theoretical basis for understanding the mechanisms through which the COVID-19 pandemic influenced stock market volatility in the Pakistan Stock Exchange.

### 2.2 Empirical literature review

Economic history shows that the stock market reaction to pandemics is always cyclical [15]. Stock market performance history has been written in many research articles, which crystallize the effect of influenza and different types of epidemics on stock market performance.

In Pakistan, [16] examined the impact of COVID-19 on Karachi Stock Exchange (KSE) and concluded that COVID-19 cases have negative impact on the performance of KSE. [17] shows insignificant impact of positive cases and deaths on the stock market performance. Therefore, their findings are opposite to the global research findings because of ignoring other factors which may affect stock market performance. Hence, these studies provide a significant gap in the existing literature to investigate the volatility pattern during crisis period with accurate method of estimations for clear conclusion.

[18] conducted a study to investigate the share market prices are related to specific events and found the significant relationship between them. According to [19] that the COVID-19 has significant negative and positive impact on the performance of organizations, and they also concluded that some companies maintained their sustainability even though most of the firms suffered from the pandemic. Moreover, [20] investigated the impact on the COVID-19 on the three different stock markets belong to different region such as Pakistan, China and the USA and found the significant negative relationship between the COVID-19 and stock market. They also concluded that the lockdown in the economy also decreased the stock market performance of the country. [21] also investigated the consequence of the COVID-19 in Pakistan at different time period and concluded the cultural challenges during the COVID-19 policy control. Therefore, these studies provide a significant gap in the literature about the stock market volatility pattern during the period of pandemic.

Similarly, equity markets have been seen for some time as important in predicting real economic movement [22]. Moreover, Stock market volatility is greatly linked with uncertainty in the stock market, which is an important factor for investment alternatives choice in any stock market and it is important and reliable risk forecaster [23]. There has been lot of evidences that financial markets have structural fractures that affect fundamental financial measures like stock returns and stock market volatility [24]. Various economic events, according to empirical evidence, cause structural changes to be observed in a large number of financial series, particularly during times of crisis [25]. Knowledge of the stochastic behavior of correlations and covariance between asset returns is critical in asset pricing, portfolio selection, and risk management in this setting [26].

[27] gives immediate research on the connection between excess returns and volatility. They note that market abundance returns are defined strictly by the normal volatility of stock returns, but negatively defined by the sudden volatility of stock returns.

According to [28], stock market performance is affected with change in the level of financial support by the government to different sectors during pandemics like COVID-19. Stock market performance is also affected by the preventive restrictions imposed by the government on different sectors like timing of opening and closing of business activities, closure of construction industry and exemption to some businesses from closure like pharmaceutical industry, etc. during lock down [29].

However, COVID-19 is a source of systematic risk; therefore, it is necessary to verify its impact on financial markets [30]. According to [25], crises have similar effects on economy as well as stock markets to great extent. [31] described five stages of the 2008 Global Financial Crises: mortgage disaster; expansion of credit risk; bad liquidity impact; the commodity price bubble; and final catastrophe of credit market. The stock market’s volatility has changed throughout time, as shown by several studies. [32] stated that variations in volatility are mostly caused by changes in macroeconomic variables. According to [33], financial leverage is a contributing factor in the occurrence of changes in volatility. Many studies have attempted to relate changes in the volatility of the stock market to changes in the anticipated returns of stocks. [34] found that stock markets are less unpredictable when the market is closed due to some reason, regardless the reason may be the lockdown due to pandemic or war. Therefore, this study addresses the gap of the risk that should be long term or short term in the period of the financial constraints that has the main problem in the emerging economy especially in the Pakistan that already faced many other macroeconomic disturbances in their economic system.

## 3. Methodology

### 3.1. Data description and sample collection

To explore the impact of COVID-19 period on stock market volatility, we used the secondary data extracted from World health organization (WHO) website (https://www.who.int/data/collections) and index data provided by the Pakistan stock exchange on their website (https://dps.psx.com.pk/) for the period 15^th^ of the March 2020 to 31^st^ March 2021. The World health organization has regional offices around the world and these offices support the national health structure in different ways. In Pakistan, world health organization worked with coordinating to the Ministry of national health services regulation and Coordination (NHSRC) to support the health facilities within Pakistan. The National command and control authority (NCCA) collect the data and monitor throughout Pakistan and provide to NHSRC. The NHRC communicates the data to the WHO for better health discussion. According to [35] that the WHO collects the data through their regional offices from the respected country health system. The data of the COVID-19 and the stock market index are collected on a daily frequency basis. Therefore, 382 total observations were used in the analysis.

The data sample selected time period is the main domain of the analysis because it covers the initial boom and the declining phase of the pandemic. Moreover, after 31 March 2021 the cases of the COVID-19 reduced to their lowest range. Pakistan stock market is selected on the phenomenon of the cultural aspect different from other emerging economies that already faced different difficulties such as political instability and the economic downfall from the last decades. While the other emerging as well as the developed economies should maintain their economic position in during the pandemics by conducting their business activities through online platform but due to lack of the resources Pakistan faced difficulties and sustain on the IMF programs.

### 3.2 Measurement and significance of the variables

The market return is extracted from the PSX 100 index of the Pakistan stock exchange. The return is calculated by the following formula,

$$\text{Return}=\left(\text{Closing}\;\text{price}\;\text{of}\;\text{index}-\text{opening}\;\text{price}\;\text{of}\;\text{index}\right)/\text{opening}\;\text{price}\;\text{of}\;\text{index}$$

According to [36] that the stock market return is useful for indicating the overall stock market performance and we can measure the risk through the return of the stock. [37] used the given formula to calculate the stock market return in their study and concluded that the stock market return is the indicator of the financial domain that leads to economy to the stage of the development with proper utilization without speculation in the market by investors. Stock market returns are inherently volatile, with prices influenced by a variety of factors such as economic news, geopolitical events, and company performance. When making investing decisions and controlling risk, investors must take volatility into account. The importance of stock market profits varies according to an investor’s time horizon. Long-term investors who are focused on attaining their financial goals over several years or decades may not be as concerned about short-term swings. The performance of one country’s stock market can have an impact on global markets. International investors constantly monitor the performance of stock markets around the world in today’s linked world, and happenings in one market can have an impact on others.

The volatility is measured by the standard deviation of the return of the stock market [38]. Moreover, greater volatility is indicated by a higher standard deviation. In the context of the stock market, increased volatility indicates that prices or returns have fluctuated more over a specific time period. Reduced standard deviation, on the other hand, signifies reduced volatility, implying more consistent and predictable returns. Standard deviation is used by investors and analysts to estimate the risk of an investment. Higher volatility is frequently connected with increased risk since it suggests greater uncertainty and the possibility of larger losses. less volatility is regarded as less dangerous, but it may result in lesser potential rewards. The standard deviation of individual equities and the market as a whole is critical for portfolio design. Investors can develop a diversified portfolio that seeks to strike a balance of risk and return by combining assets with different volatility profiles. Moreover, we used the period of the high active cases from beginning to its declining stage in our study.

### 3.3 Models improvement and description

According to the [39] that ARCH model has the one drawback that work like the moving average instead of autoregression. From this new concept, which includes the lagged conditional variance term used as the autoregressive term. This concept was developed by the [40] for the first time in his paper and generated the new concept in Family of GARCH model. According to [40] that GARCH (p, q) model concept is based on a phenomenon that conditional variance of a time series depends on the squared residuals. It is possible to estimate heteroscedasticity by using the GARCH model specifications. [40] shows that all GARCH models are martingale difference models, all expectations are erroneous. As a result, the GARCH (p, q) model can be viewed as a simplified variant of a more sophisticated dynamic structure for time-varying conditional second order moments. In order to determine the tendency for clustering of volatility, it is possible to analyses financial data using GARCH models. According to [41], A GARCH model’s conditional mean, is stated as an explicit function of condition variance. GARCH-M is the name given to this type of model. The GARCH (p,q)-M Model can be used to represent stock returns. A significant instrument in asset pricing and financial risk management, the GARCH family of volatility models has emerged since then. Various econometric studies have been conducted on volatility estimate and forecasting the work of [41–43]. Moreover, with the addition of the ARCH models, others GARCH models such as GARCH-Means Model, IGARCH model, Threshold GARCH models are used to capture the stock volatility in different time period.

In order to increase the GARCH model’s ability to capture return properties, alternative models were developed. On the other hand, the optimal model for capturing volatility has not been determined in previous studies. Simple GARCH (p,q) models have been found to be more effective in some studies than more complex ones. Each model has its own performance characteristics that are dependent on the market and usage conditions. The measurement of the error terms is the main drawback of these forecasting models that should be improved with respect to time.

Our goal is to find the most accurate model for Pakistani stock market. Two models, one symmetric and one asymmetric, will be compared (EGARCH and TGARCH). We used the GARCH methodology on the grounds of measuring the short- and long-term effects of the risk on the stock market especially in the period of the COVID-19. GARCH model is suitable because it captured the variance in the time series data. Through the variance fluctuation, we can measure the effects of the risk on the return of the stock market, but the other methods do not capture the short and long run behavior of the volatility. Financial institutions, portfolio managers, and individual investors can use GARCH models to assess and manage risk. These models enhance risk management methods by offering projections of future volatility, allowing investors to make informed decisions about asset allocation and position sizing.

Volatility clustering, as captured by GARCH modeling, is one of the specific characteristics of stock market returns. Therefore, we use the following GARCH (1,1) model to estimate time-varying volatility for *r*_*t*_, a country’s stock market return:

$$r_{t}=\alpha +\beta r_{t-1}+\epsilon_{t}\;\text{where,}\;\epsilon_{t}|I_{t}\sim N\left(0,\sigma_{t}^{2}\right)$$ (1)

and

$$\sigma_{t}^{2}=\omega_{0}+\omega_{1}\epsilon_{t-1}^{2}+\omega_{2}\sigma_{t-1}^{2}.$$ (2)

Eq (1) indicates the average model equation while Eq (2) indicates the conditional uncertainty that tracks transient fluctuations of the stock market, capturing the conditional volatility that capsulate the time-variable uncertainties in the financial markets of our study.

[44] used daily stock price data from January 2006 to April 2011 to examine the impact of the financial crisis on different economies such as China, Japan, India and US stock market. The subject of stock market volatility is extensive. Empirical studies utilizing GARCH and ARCH models capture the stock market’s volatility.

According to a number of studies, researchers have discovered that GARCH family models are the most accurate when it comes to predicting stock market volatility [45]. These models are useful for conditional distributions of the tail thickness and also shows the importance of the skewness of the return. The Fat-tailed density measured with the help of the asymmetric GARCH model improved the conditional variance estimation.

The Generalized Autoregressive Conditional Heteroscedasticity model referred as GARCH was developed from the foundations of the ARCH for the first time [46]. The univariate GARCH models are not appropriate for many analyses due to the assumption of the volatility’s constant over some period of time among the variables. Univariate GARCH does not captured the volatility among multiple time series data [47]. Dynamic correlations are not also captured but it only captures the linear correlation. This gap should be filled by the constant conditional correlation CCC- GARCH model, but it also has the weakness of detecting the dynamic correlation. To detect the dynamic correlation on different time domain [46] developed the model based on the constant conditional correlation model.

For our study we selected the DCC-GARCH model that is developed by the [46] that is useful for the time varying volatility and detecting the correlation between the stock markets and the COVID-19 cases. The [46] model is based on the Gaussians distribution that is not a proper method for the different time series or heavy tailed distribution but [47] used a model that is Multivariate distribution called DCC-GARCH method that is suitable for the multiple time series.The general Equation of the DCC-GARCH are given below,

$$H_{t}=D_{t}R_{t}D_{t}$$

In this equation *H*_*t*_ represents the conditional variance and where *D*_*t*_ represents the diagonal matrix that having conditional variance, *R*_*t*_ is the time varying correlation matrix. The conditional variance for the Assets that represents *H*_*t*_ are estimated firstly by univariate GARCH (X, Y) model. The *D*_*t*_ matrix can be represented by $D_{t}=diag\left(\sqrt{h_{t}^{x}},\sqrt{h_{t}^{y}}\right)$, that is used for the conditional standard deviation of the time series t, that function obtained from the by univariate GARCH (X, Y) model that is given below,

$$h_{t}=c+ae_{t-1}^{2}+bh_{t-1}$$

In above equation c represents the constant with *h*_*t*_ is denoted the conditional variance, with *a* and *b* two different parameters that is useful for capturing the ARCH and GARCH effect. Time varying conditional correlation is represented by *R*_*t*_ = [*ρ*_*xy*,*t*_] matrix.


$$R_{t}=diag{\left\{Q_{t}\right\}}^{-1}Q_{t}\;diag{\left\{Q_{t}\right\}}^{-1}$$

In the above equation unconditional correlation is represented by the function *Q*_*t*_ = [*q*_*xy*,*t*_] for the *e*_*t*_ matrix. The time-varying correlation estimator is extracted by calculating:

$$Q_{t}=\left(1-\alpha -\beta \right)\bar{Q}+\alpha e_{t-1}e_{t-1}^{\prime }+\beta Q_{t-1}$$

$$\rho_{xy,t}=\frac{q_{xy,t}}{\left(\sqrt{q_{x,t}},\sqrt{q_{x,t}}\right)}$$

In the above equation $\bar{Q}$ is used for the unconditional correlation of the standardized residuals and model means reverting if *α* + <1.

#### 3.3.1 Time varying volatility

As per the GARCH modeling, volatility clustering is one of the specific characteristics of the stock market return. Before the volatility analysis through GARCH Modeling, we should have to fulfil the GARCH assumption of the volatility clustering existing in the stock market return. Therefore, we use the GARCH (1,1) model to estimate the time varying volatility for *r*_*t*_, a country’s stock market return:

$$r_{t}=\alpha +\beta r_{t-1}+\epsilon_{t}\;\text{where,}\;\epsilon_{t}|I_{t}\sim N\left(0,\sigma_{t}^{2}\right)$$ (3)

$$\sigma_{t}^{2}=\omega_{0}+\omega_{1}\epsilon_{t-1}^{2}+\omega_{2}\sigma_{t-1}^{2}.$$ (4)

Eq (3) indicates the average model equation, while Eq (4) indicates the conditional uncertainty that tracks transient fluctuations of the stock market, capturing the conditional volatility that capsulate the time-variable uncertainties in the financial market of our study. Our goal is to analyses both co-movement between stock market return and the COVID-19 cases. Therefore, to attain our objectives of the study, we used the above discussed methods of the estimations for drawing the conclusion of the study.

## 4. Results and findings

The descriptive statistics in Table 1 shows that the average daily active cases of 1086 with maximum 6884 and minimum 0 and the stock price has means value 39138 index value in Pakistan stock exchange with maximum of 46091 and minimum 27228 in the selected period. The average return of the stock market is -0.00043 with a maximum of 0.073607 and minimum of -0.04576. in the 307 days data for Pakistan. Higher volatility is being observed in the selected period due to the pandemic effects. There is week correlation existed in the study variables as shown in Table 2.

**Table 1:** Descriptive statistics.

Descriptive	COVID	CV	R
Mean	1086.254	39138.9	-0.00043
Median	566	40504.75	-0.00124
Maximum	6884	46091.96	0.073607
Minimum	0	27228.8	-0.04576
Std. Dev.	1463.676	4151.242	0.014531
Skewness	1.90731	-0.77499	1.279061
Kurtosis	6.096823	2.788812	9.377529
Jarque-Bera	308.8118	31.30169	603.9825
Probability	0	0	0
Sum	333480	12015643	-0.13086
Observations	307	307	307

Source: Author computations.

**Table 2:** Correlation matrix.

	COVID	CV	R
COVID	1		
CV	0.207889	1	
R	-0.05429	0.022761	1

Source: Author computations.

The volatility clustering among the COVID-19 cases, closing value of the stock and returns are shown in Fig 1. Preliminary tests have been conducted to support the suitability of the GARCH family and wavelet methodology, which include the Augmented Dickey Fuller Test, assessment of ARCH effect, and examination of volatility clustering in the data [48]. The results of Preliminary tests are summarized in Table 3. The ADF test provides insights into the data’s stationarity, while the Chi-squared value from the ARCH effect indicates the presence of ARCH effect and its compatibility with GARCH volatility. Fig 1 helps to determine the presence of volatility clustering in returns.

**Fig 1:** Volatility clustering.

**Table 3:** Prerequisites test for GARCH.

COUNTRY	ADF	Chi- squared
PAKISTAN	-19.712***	744.90***

Note: In ADF and Chi- squared level of significance is 1%, 5% and 10% representing ***, ** and * respectively.

Source: Author computations.

Our findings reveal that the ADF values for the return series are statistically significant at a 1% level, implying that the data exhibits stationarity after differencing and is suitable for analysis using the GARCH and wavelet approaches. The Chi-square value is also significant for Pakistan, indicating the presence of ARCH effect in the stock market returns, which is crucial for GARCH family models. The graphical representations clearly demonstrate that small changes in returns are followed by small changes, while large changes are followed by large changes in the stock market returns of Pakistan. This observation confirms the fulfillment of the volatility existence assumption before applying the GARCH volatility model. If all these preliminary tests yield statistically significant results, we can proceed with the analysis using GARCH, which will provide more accurate and reliable conclusions.

The lag selection is based on vector autoregressive (VAR) model. We select the lag value that is 2 and that’s why our GARCH estimation is (2,2). According to the [49] that the lag selection should be done based on Schwarz information criterion (SC) and Hannan-Quinn information criterion (HQ), when both parameters are significant at same point and less lag is suitable for the accurate result. Lag selection in econometrics is a critical point due to the different opinions of the research and previous research done on lag selection. Below Table 4 represents the lag selection criteria.

**Table 4:** VAR lag selection criteria.

*Lag*	*Log L*	*LR*	*FPE*	*AIC*	*SC*	*HQ*
0	-4669.12	NA	7.50E+09	31.25162	31.28875	31.26648
1	-3514.21	2278.918	3516758	23.58668	23.73519*	23.64612
2	-3496.32	34.94143*	3313811.*	23.52721*	23.78711	23.63124*
3	-3488.1	15.87919	3331436	23.53247	23.90375	23.68107
4	-3486.57	2.941168	3502265	23.58239	24.06505	23.77557
5	-3482.42	7.853209	3618296	23.61484	24.20889	23.8526
6	-3480.84	2.949573	3803330	23.6645	24.36994	23.94685
7	-3479.5	2.483055	4004419	23.71574	24.53256	24.04267
8	-3474.75	8.71971	4121224	23.74412	24.67232	24.11563

Source: Author computations

Note. Lag order Selection criteria on the basis of the VAR model are given above, were the

* Indicates lag order selected by the criterion

LR: sequential modified LR test statistic (each test at 5% level)

FPE: Final prediction error

AIC: Akaike information criterion

SC: Schwarz information criterion

HQ: Hannan-Quinn information criterion

### 4.3 GARCH volatility

In the given Table 5, the output of univariate exponential generalized autoregressive conditional heteroscedastic (E-GARCH) to estimate the volatility for stock market and other factors are given. Univariate GARCH is very useful to estimate the Volatility in each stock market and selected variables individually. The Univariate GARCH values are estimated on the basis of the E- GARCH that is given in table with means and variance equation. First Columns indicated the coefficient The ARCH term (ω1) (also known ARCH Alpha) is also significant, it means that short term volatility is found in Pakistan Stock return, while GARCH term (ω2) (also known as GARCH Beta value) is also statistically significant, it means that persistent of volatility in the Pakistan stock market exist for the long run. Hence, the sum of both ARCH and GARCH term is also large, indicating the effect of the shock remains in forecasting variance for long period of time in the future. coefficient for the mean equation, while the second column is related to the variance equation. In our estimated model of the E-GARCH all the values of the ARCH alpha and GARCH beta are significant, indicating that there is both short term and persistent volatility in all selected variables found for long run.

**Table 5:** E-GARCH findings.

**Mean Equation**						
	Constant(α)		P-Value	Lag (1) (β)	P-value	
Return	0.0203		0.0000***	0.1145	0.0000***	
CV stock	0.0565		0.0000***	-0.0089	0.0000***	
Cases	0.0638		0.0000***	-0.0141	0.0000***	
**Variance Equation**						
	Constant (ω)	P-value	ARCH (1) (ω1)	P-value	GARCH (1) (ω2)	P-value
Return	0.0051	0.0000****	0.0896	0.0000	0.9112	0.0000***
CV stock	0.0239	0.0000****	0.0884	0.0000	0.8976	0.0000***
Cases	0.0242	0.0000****	0.0903	0.0000	0.8961	0.0000***

Source: Author computations

Various news, events, and incidents can impact investors’ decision-making processes. When making investments, investors consider these factors as a primary consideration. These events, news, and incidents have an asymmetric impact on financial markets. Mergers, acquisitions, and trade partnerships also influence investors’ decisions and significantly affect financial markets. Consequently, the impact of positive and negative news differs and may exhibit asymmetry. Sometimes, negative news has a greater impact than positive news, and vice versa.

In this analysis, we introduce the term Gamma (ѱ) to capture the asymmetric impact of good and bad news on the stock market, taking into account the leverage effect. We also examine the persistence in volatility, which should be less than 1, including ω1+ω2+ ѱ/2. If the Gamma (ѱ) value is statistically significant and positive, it indicates that a negative shock will lead to a greater increase in volatility than a positive shock. Based on the following points, we can conclude that in the asymmetric GARCH model, a negative shock results in higher volatility compared to a positive shock.

Our results reveal that the Gamma (ѱ) value for the stock market is positive and statistically significant at a 1% level of significance. This implies that negative shocks increase volatility more significantly than positive shocks. Essentially, this suggests that during a market crisis, volatility increases to a greater extent, adversely affecting the economy. Threshold (T-GARCH) results are presented in Table 6.

**Table 6:** Threshold GARCH results.

T-GARCH			
	ARCH (1) (ω1)	GARCH (1) (ω2)	Gamma (ѱ)
Pakistan	0.3019***	0.7152**	0.1823***

Note: The Variance equation is: $\sigma_{t}^{2}=\omega_{0}+\omega_{1}\epsilon_{t-1}^{2}+\omega_{2}\sigma_{t-1}^{2}.\;r_{t}$ represents the stock return of a particular country. The level of significance is 1%, 5%, and 10%, respectively

Source: Author computations

Multivariate analysis occurs when one univariate time series impacts another univariate time series. Similarly, if the stock market in different regions experiences an influence from COVID-19 cases, we can infer the existence of a multivariate relationship between them. To examine the relationship between volatilities and co-volatilities among multiple univariate stock markets and COVID-19 cases, we can employ the Multivariate GARCH model. A specific type of Multivariate GARCH methodology is the DCC GARCH model, which focuses on determining the correlation between volatilities in two time series. In this study, we opted for the DCC GARCH model because it directly parametrizes the conditional correlation. It considers the interdependence of one stock market on the prevailing conditions in the environment. The Dynamic Conditional Correlation GARCH (DCC-GARCH) model captures the relationship between two or more variables that rely on past information and vary over time, rather than remaining constant. The DCC-GARCH model quantifies the conditional correlation through two parameters: DCC Alpha (γ1) and DCC Beta (γ2). Both γ1 and γ2 signify the dynamic and time-varying behavior captured by the estimated model. DCC Alpha (γ1) describes the short-term volatility impact from one time series to another, indicating the persistence in the standard residual from the previous period. On the other hand, DCC Beta (γ2) measures the lingering effect of shocks, representing the persistence of conditional correlation within the model. The sum of these two parameters should be less than one, indicating that the conditional correlation in the model does not remain constant over time and exhibits dynamic behavior. Table 7 represents the DCC-GARCH findings of spillover effects.

**Table 7:** Spillover effect of COVID-19 cases on stock market return volatility.

Pair	DDC Alpha (γ1)	P-value	DCC Beta (γ2)	P-value
COVID-Return	0.01192***	0.0000	0.7892***	0.0000

Note. The level of significance is 1%, 5%, and 10%, representing ***, ** and * respectively.

Source: Author computations

Similarly, if the DDC Alpha (γ1) value is found to be statistically insignificant, it implies that there is no short-term persistence observed between the two-time series. Conversely, if DCC Beta (γ2) is significant, it suggests the presence of long-term persistence between the two-time series. In our findings, when examining the relationship between COVID-19 daily cases and the stock market returns in Pakistan, we observe that DDC Alpha (γ1) is statistically significant. This signifies the existence of a short-term spillover impact of COVID-19 cases on the stock market of Pakistan. Additionally, DCC Beta (γ2) is also significant in this pair, indicating a long-term spillover impact of the pandemic on return volatility.

## 5. Discussion on findings

In our findings, there is both short term and persistence in volatility for long run found in the stock market return of Pakistan during the period of pandemic. The presence of both short-term and persistent volatility in the stock market returns of Pakistan during the pandemic period can be attributed to a combination of factors. In the short term, the sudden onset of the pandemic led to widespread uncertainty and panic selling, causing sharp market fluctuations. These short-term bursts of volatility were driven by factors such as rapidly changing information about the pandemic’s impact on the economy, government policy responses, and global market sentiment. In the long run, persistent volatility can be explained by ongoing economic and geopolitical uncertainties, as well as concerns about the pandemic’s prolonged effects on various sectors of the economy. Additionally, structural weaknesses within the Pakistani economy and financial system may have contributed to long-term volatility. These combined factors created a complex interplay of short-term and persistent volatility in the stock market, making it a challenging environment for investors and reflecting the broader economic and geopolitical uncertainties associated with the pandemic. Therefore, our findings are similar directions with the previous study by [50] but our study add in this study by including all type of fluctuation related to the boom, decline in the COVID-19 cases and find the both short and long run volatility but [50] found only the short term.

Our results reveal that negative shocks increase volatility more significantly than positive shocks. Essentially, this suggests that during a market crisis, volatility increases to a greater extent, adversely affecting the economy. The greater impact of negative shocks on increasing volatility during a market crisis can be attributed to a combination of psychological factors, market dynamics, and systemic vulnerabilities. Investors tend to exhibit heightened sensitivity to adverse news, as loss aversion leads to more rapid and pronounced reactions to negative developments. Liquidity concerns often arise during crises, making it easier for negative shocks to trigger panic selling and sharp price declines. Additionally, negative shocks are often associated with systemic risks that raise concerns about the stability of the financial system, further amplifying market reactions. The adverse effects of increased volatility during a crisis ripple through the economy, eroding investor and consumer confidence, tightening credit conditions, and necessitating more significant policy responses. This asymmetric response to shocks underscores the fragility of financial markets and the interconnectedness between market behavior and broader economic well-being during times of crisis. In this way our findings are similar with the previous findings by [51] that reveal the asymmetric effect of the COVID-19 news on the market.

In our findings, there is both short-term and long-term spillover impact of COVID-19 cases on the stock market of Pakistan. The occurrence of both short-term and long-term spillover effects of COVID-19 cases on Pakistan’s stock market explained by the pandemic’s varied effects on financial markets. In the short term, this study has revealed that markets are very responsive to daily swings in COVID-19 cases, reacting to news regarding infection rates, lockdown measures, and vaccine advances and our findings are similar with previous literature of [52]. Long-term stock market effects of the pandemic include interrupted supply chains`, fluctuations in consumer behavior`, and structural changes in businesses [53]. Even after the current health crisis has passed, these factors continue to have an impact on business profitability and market performance [54]. As a result, the observed spillover effects on Pakistan’s stock market are the result of a combination of short-term sentiment-driven reactions and long-term structural changes in the aftermath of the pandemic.

## 6. Conclusion and recommendation

Our first objective is to investigate the volatility pattern in stock market return during the period of COVID-19 pandemic. Related to our objective, our findings show the during the selected period of pandemic period at different stages Pakistan stock return has both short term volatility pattern and also found the long-term persistency in their volatility due to long term effects of the cOVID-19 cases through Pakistan. The persistency in the return volatility indicated the lockdown due to the fear of spread of COVID-19 cases that leads the high risk in the market. The spread of the risk may be different in each economy around the globe due to different measures and the strength of the financial system in the country.

Our second objective was to investigate the impact of the news spread in the economy about the disease on the stock market in Pakistan. Related to this objective, our findings show that the bad news in the market has greater effect as compared with the good news to fear and other factors. Our third objective was to investigate the change in the volatility of the return due to the change in the COVID-19 cases. In this way, our results demonstrate the presence of both short-term and long-term spillover effects that indicate the influence of the COVID-19 pandemics on the stock market return and create negative consequences for the overall economic growth of the country. There are many reasons behind the consequences, the most significant reason is the lockdown of the business activities that create the risk for the stock market and its stakeholders [55]. Therefore, these findings emphasize the importance of considering external factors, such as COVID-19 cases, when analyzing stock market behavior. Investors and analysts should be aware of the potential linkages between pandemics and financial markets, as they can significantly impact investment decisions and overall market performance. Moreover, it is worth noting that the results are specific to the case of Pakistan and may not be directly applicable to other countries or regions. Factors such as local economic conditions, government policies, and market dynamics can influence the relationship between COVID-19 cases and stock market returns differently in various contexts.

### Policy implication and suggestion for future research

The study has several implications for investors, government and policy makers. Investors can manage their risk taking the volatility pattern of the respected country in mind. The volatility and spillover are useful for the investor to keep in mind while making the internationally diversified portfolio for getting the expected rate of return especially in the distress time period. This study is also helpful for investors to raise investor confidence by seeing the pattern of the volatility in the period of the pandemic. Generally, investors prefer low volatility stock during the distress period and like high volatility stock at normal period [56].

The study also provides implications for policymakers about the effectiveness of various policy interventions implemented during the pandemic to stabilize the stock market. Governments and regulatory bodies can assess the impact of fiscal and monetary policies, market regulations, and stimulus measures on market volatility. The findings can guide policymakers in formulating appropriate measures to support the market and investor confidence during future crises. Understanding the differential impacts of the pandemic on various sectors of the Pakistan Stock Exchange can have implications for investors, industry participants, and policymakers.

Moreover, examining the long-term effects of the pandemic on stock market volatility can have implications for the overall market structure and dynamics. The findings can help in identifying structural shifts or changes in investor behavior that may persist beyond the pandemic which is valuable for market participants and policymakers in anticipating and adapting to potential future disruptions.

To analyzing the effect of the COVID-19 on all Asian and OECD economy is the difficult task due to the limitations and open the door for the new insight for further research to investigate on all Asian and OECD economy for different culture comparison. Moreover, pre-and post- pandemic behavior of volatility should be the future research topic for investigation especially in the merging economy where every country struggles to increase their economic sustainability. Future research may be conducted on the different economic indicators such as inflation, interest rate, unemployment and government expenditure should be included with COVID-19 cases for getting volatility pattern. Moreover, governance mechanism in the country may contribute in raising the effects of the pandemic on the stock market return, it may be investigated in future research topic.

## Supporting information

S1 Data Pak return and covid. (XLSX)
